# Boundary Determination of Lake-Type Wetland Park Based on GIS Multifactor Analysis

**DOI:** 10.1155/2022/6161491

**Published:** 2022-06-06

**Authors:** Guodong Chen, Peng Tang, Hao Wang

**Affiliations:** ^1^College of Landscape Architecture, Nanjing Forestry University, Nanjing 210037, China; ^2^College of Environmental Ecology, Jiangsu Open University, Nanjing 210017, China

## Abstract

One key carrier for wetland resource protection is wetland park, the main form of which includes lake-type wetland park. To determine the management and control boundary of lake-type wetland parks scientifically and reasonably is of great significance to the sustainable protection and utilization of wetland resources. From the perspective of landscape architecture, and landscape ecology, this paper studies the boundary determination of Changdang Lake National Wetland Park (the Park) based on satellite remote sensing information technology and GIS technology and in virtue of Analytic Hierarchy Process (AHP). In this study, 12 subindicators were selected from three levels including visual control, human geography, and ecological control. The weight of each indicator was determined by AHP, and then the influencing factors were transformed into graphic data by using GIS technology. Finally, the Park's boundary was determined by factor superposition analysis based on the weight. The research shows that the newly defined management and control boundary are about 340 sq.km, which effectively integrates the human and natural ecological resources around the lake area, makes the development of the surrounding areas harmonious, ensures the integrity of the lake area ecosystem, and facilitates the sustainable development of wetland resources.

## 1. Introduction

As a kind of important ecological strategic resource for human's sustainable development, wetland is hailed as “the kidney of the Earth” thanks to its outstanding function for ecological environment regulation and ecological benefit. In the face of deterioration of natural environment and human activities threat, to strengthen the protection and sustainable utilization of wetland resources has become the shared idea of the wetland circle worldwide [1]. As a combination of wetland protection, ecological restoration and sustainable utilization of wetland resources, wetland park can alleviate wetland resource loss effectively [2], and shall be managed and protected on the basis of determining the management and control boundary scientifically and reasonably [3].

Without a clear concept of “wetland park”, European and American countries study the wetland mainly relying on the “natural wetland and artificial wetland in national parks” and therefore have not specifically studied the boundary determination of “wetland park” protection [4]. Their research on the boundary mainly focuses on the wetland ecosystem [5]. Vegetation, soil, and hydrology are the most commonly recognized important characteristics of wetland ecosystem. Researchers studied the determination of wetland boundary by studying the 13 marine wetlands in Oregon and Washington, coastal wetlands in San Quentin, California, pine wetlands in New Jersey, cypress wetlands in Florida, everglades wetlands in Virginia/North Carolina, and coastal wetlands in South Carolina using on one, two or all of the three indicators above since the 1970s [6].

China started individualized study on “wetland park” since the beginning of the twenty-first century. At present, the boundary of “wetland park” is determined mainly in the form of “ecological redline” [7, 8], which was clearly put forward in the Opinions of the State Council on Strengthening the Key Work of Environmental Protection in 2011: the ecological redline shall be defined in major ecological functional areas, sensitive areas of land and marine ecological environment, vulnerable areas, etc. As the boundary line, and management and control line of the ecological area, the ecological redline can cope with the environmental resources constraint pressure ascribed to China's rapid urbanization process effectively and maintain national or regional ecological security and sustainable development, enabling its application to wetland park [9]. Lake-type wetland park is the main type of China's wetland parks. As a kind of important wetland resource, lake plays an irreplaceable role in maintaining biodiversity, conserving water resources, regulating climate, and promoting the sustainable development of regional ecological economy [10]. At present, the redline determination of lake-type wetland park is actually dominated by the government alone. For the sake of management and implementation, the whole lake or some lake surface and related areas are selected as the redline range of wetland park in the principle of ecosystem integrity and uniqueness to carry out functional zoning and put forward the specific protection and restoration measures [11].

Some important aspects for the present research on the protection and utilization of lake-type wetland park are the following: how to explore a boundary determination method that can not only coordinates the ecological safety of the whole lake basin but also meets the functional requirements of ecotourism, publicity, education, and scientific research of wetland park. How to improve the scientificity and operability of the lake wetland boundary determination and control lake ecosystem dynamically. How to form a set of boundary determination system with universal significance and applicable to lake-type wetland park.

With the rapid development of information technology since the 1990s, GIS technology has been widely applicable to landscape ecology and landscape architecture. GIS technology, featured by strong ability of spatial analysis and data processing, can hardly determine the index weight of each influencing factor. Therefore, AHP is introduced in this paper to determine the index weight. AHP, which was first proposed by Professor T.L. Saaty, an American operational research scientist in the early 1970s, is used to solve complex multiobjective decision-making problems. The decision-making problem can be broken down into target layer, criterion layer, factor layer, etc. By comparing two pairs of scale values, the judgment matrix is constructed and the qualitative problem that people judge via subjective experience is quantified, which greatly enhances the order and scientificity of decision-making [12]. The influencing factors of boundary determination of lake-type wetland park are analyzed quantitatively by GIS technology and in virtue of the advantages of GIS technology and AHP, and then are transformed into graphic data to establish a buffer zone and form a plane graphic state; finally, factor superposition analysis is carried out according to the weight of each influencing factor determined by AHP, so as to get the final wetland park protection boundary. To determine the protection boundary based on the GIS technology, AHP can make up for the shortcomings and limitations of the traditional boundary determination effectively. The combination of qualitative and quantitative analysis ensures the scientificity and operability of the boundary determination.

Main objectives of this study:

1. Build boundary determination system of lake wetland based on AHP and GIS spatial analysis technology from the perspective of landscape ecology and landscape architecture by taking Changdang Lake National Wetland Park as an example.
2. Determine the management and control boundary of the Park.
3. Provide basis for the protection and sustainable utilization of wetland resources.

## 2. Research Area and Data

### 2.1. Research Area

Changdang Lake, located in Changzhou City, Jiangsu Province, China, spans Jintan District and Liyang City in Changzhou. It is 9 km far away from the southeast of Jintan and 20 km from the northeast of Liyang City (Figure 1). There are many canals, ditches, and rivers as well as mountains within the scope of Changdang Lake basin featured by extremely abundant habitat types and giving birth to rich wetland biological resources and wetland landscape resources. As an important regulation and storage lake between the Yangtze River and Taihu Lake, Changdang Lake has stable wetland ecosystem structure and healthy wetland functions, which are of great significance to water environment safety and wetland resource protection of the Taihu Lake basin.

To protect the wetland resources of Changdang Lake more comprehensively, Jintan district government launched the planning and construction of the Park, which has a total planning area of about 76.9 sq.km, including 72 sq.km. Lake body and main river water area covers lake wetland, swamp wetland, lakeside damaged wetland (aquaculture area), and some land area administrated by Jintan district. The above brings dramatic exemplary significance for the restoration and conservation of lake wetland around Taihu Lake basin [13].

### 2.2. Current Situation of Research Region Boundary Determination

#### 2.2.1. Boundary Determination Based Water Surface, Road, and Farmland

The eastern, northern, and western sides of the Park are mainly bordered by the Yingfeng River besides Changdang Lake, its northwest side is separated by Changdang Lake West Road, and some of the western part is bordered by polder and ridge (Figure 2). Based on the terrain and features of the substance, this method overemphasizes the static management and control of the wetland park and ignores the dynamic supervision of the lake basin ecosystem. Some river water networks along the lake are not included in the management and control scope of the wetland park, and enough ecological buffer area cannot be ensured. Some potential natural and human ecological resources along the lake are not taken in the scope of protection [14], which breaks the internal balance of the wetland ecosystem of Changdang Lake, exerts adverse influence on the sustainable development of the wetland park ecosystem of Changdang Lake, and hardly maximizes the ecological, social, and economic benefits.

#### 2.2.2. Boundary Determination Based on Administrative Boundary

The southern side of the Park is bordered by the administrative boundary between Jintan district and Liyang city. At present, the Park's water area accounts for 85% of the total area of Changdang Lake, and the rest falls into the scope administrated by Liyang city.

### 2.3. Source

Land cover information was extracted by using 2018 Landsat-8 remote sensing image (source: http: gscloud.cn). On the basis of fusion, correction, and registration of Landsat-8 remote sensing image, land-use properties were extracted by feature recognition through GIS. Data such as slope and elevation data were from DEM, the data of which are from geospatial data cloud.

## 3. Method

### 3.1. AHP Analysis Method

#### 3.1.1. Indicator Selection

This paper builds index system from visual control, human geography, and ecological control by referring to relevant literature on the study on boundary determination such as natural reserves, world cultural and natural heritage, scenic spots, forest parks, geoparks and drinking water conservation areas, boundary influence factors of relatively mature boundary, and wetland [15], considering the characteristics of lake-type wetland park and according to the Park's realities and availability of data sources. Finally, the boundary determination system of lake-type wetland park includes 3 project layers and 12 index layers (Table 1) and 2.

#### 3.1.2. Determination of Index Weight

AHP method is mainly used to determine the index weight [16]. In this study, 20 experts specialized in relevant fields were mainly invited, including experts engaged in wetland landscape planning and ecological protection and local officials to give weight to each factor. The specific operation process is as follows:

(1) Determine the relative importance of each factor by using the expert scoring method through investigating the realities carefully and in detail. The 1–9 scale method was used for evaluation (Table 2).
(2) Satisfy the following requirements to construct the judgment matrix A: (i) *aij* > 0, (ii) *aji* = 1/*aij*, (*i*, *j* = 1, 2, ..., *n*). If the importance ratio of factor *i* to factor *j* is *aij*, then the importance ratio of factor *j* to factor *i* is *aji* = 1/*aij.*
(3) Acquire the maximum eigenvalue of A, that is, *λ*max (*M*) = *n*, and its corresponding feature vector is *ω* = (*ω*1, *ω*2, *ω*3, ... *ωn*) *T.*
(4) Use AHP software Yaahp to calculate the weight value of each evaluation factor.
(5) Check the consistency of the judgment matrix by the following formula:
  (1) $$\begin{array}{c} RC=\frac{IC}{IR}. \end{array}$$

If the CR is less than 0.10, it is considered that the consistency of the judgment matrix is acceptable. Otherwise, the judgment matrix should be modified properly. If the CR is greater than 0.10, the data will not produce meaningful results unless they are reexamined and judged. The table of final factor weights in this study is as follows (Table 3).

#### 3.1.3. Index Factor Grading Standard

The 12 index factors that have been determined are classified by considering the Park's realities and referring to relevant literature and the opinions of the experts above. The five-level classification standard is adopted here [17], with the specific five levels, respectively, represented by values 1, 2, 3, 4, and 5. The smaller the value is, the more this area should be included in the Park's protection boundary. See Table 3 for the specific classification standards (Table 3).

### 3.2. GIS Data Analysis and Preprocessing

The following four data processing methods are mainly used in this study. See Figure 3 for the specific analysis results.

#### 3.2.1. DEM Data Processing

Download DEM data from geospatial data cloud and use the surface analysis tool in Arc GIS10.1 to obtain evaluation, slope, and elevation analysis. Calculate and analyze the obtained data of Changdang Lake area and convert them into elevation map [18].

#### 3.2.2. Remote Sensing Image Data Processing

After remote sensing image preprocessing, obtain land-use classification by combining supervision classification and field investigation by using the MSS (4, 5, 7) band composite image. For the purpose of distinguishing forest, shrub, and grass through the multispectral image processing, the combined image of MSS (5, 6, 7) band is needed to obtain vegetation information.

#### 3.2.3. Analysis Data of GIS Buffer Zone

Establish different buffer distances for such factors as scene source, road traffic, water area based on the classification standard of evaluation factors by choosing “analysis tool,” “domain analysis,” “buffer zone,” in Arctoolbox and getting the buffer zones such as scene source, road, water area by inputting the buffer distance.

#### 3.2.4. GIS Factor Superposition Analysis

Superpose the multiple factors of the three subitems, that is, geography, ecological control, and visual control by selecting “spatial analysis tool,” “superposition analysis,” “weighted sum,” “input grid and weight” in Arctoolbox to get three results of human geography, ecological control, and visual control (Figure 4). Then superpose the results of the three items to get the final analysis results.

### 3.3. Boundary Determination Model of Lake-type Wetland Park

The boundary determination system of lake-type wetland park is constructed via Arc GIS spatial superposition analysis tool according to the Park's boundary determination index system and the weight of each factor [19–21]. The calculation formula of suitability index for boundary determination:

(2) $$\begin{array}{c} B=\sum Wi\times Xi, \end{array}$$

where *B* represents the suitability index of boundary determination, *W* represents the weight of index factor *i*, and *X* represents the suitability value of index factor *i*.

### 3.4. AHP Calculation Steps

Analytic Hierarchy Process, or AHP for short, refers to a decision-making method that decomposes elements that are always related to decision-making into goals, criteria, and plans, and then conducts qualitative and quantitative analysis on this basis. Build a hierarchy model. The goal of decision-making, the factors considered (decision-making criteria), and the decision-making object are divided into the highest level, the middle level, and the lowest level according to the relationship between them, and a hierarchical structure diagram is drawn. The highest level refers to the purpose of the decision and the problem to be solved. The lowest level refers to the alternatives at the time of the decision. The middle layer refers to the factors considered and the criteria for decision-making. For two adjacent layers, the upper layer is called the target layer, and the lower layer is the factor layer. Construct a judgment matrix. When determining the weights between factors at each level, if it is only a qualitative result, it is often not easy to be accepted by others. Therefore, the consistent matrix method is proposed, that is, all factors are not compared together, but they are compared with each other. At this time, relative scales are used to minimize the difficulty of comparing factors with different properties, so as to improve accuracy. For example, for a certain criterion, make a pairwise comparison of the schemes under it, and evaluate the grades according to their degree of importance. The judgment matrix has the following properties:

(3) $$\begin{array}{c} a_{ij}=\frac{1}{a_{ij}}. \end{array}$$

Since *λ* continuously depends on aij, the larger *λ* is than *n*, the more serious the inconsistency of *A* is. The consistency index is calculated by CI. The smaller the CI, the greater the consistency. The eigenvector corresponding to the largest eigenvalue is used as the weight vector of the influence degree of the compared factor on a certain factor in the upper layer. The greater the inconsistency, the greater the judgment error caused. Therefore, the inconsistency of *A* can be measured by the value of *λ*−*n*. The consistency index is defined as follows:

(4) $$\begin{array}{c} CI=\frac{\lambda -n}{n-1}. \end{array}$$

*CI* = 0, there is complete consistency; *CI* is close to 0, there is satisfactory consistency; the larger the *CI*, the more serious the inconsistency. To measure the size of *CI*, the random consistency indicator *RI* is introduced:

(5) $$\begin{array}{c} RI=\frac{CI_{1}+CI_{2}+\cdots +CI_{n}}{n}. \end{array}$$

Among them, the random consistency index *RI* is related to the order of the judgment matrix. In general, the larger the order of the matrix, the greater the possibility of random deviation of consistency.

Considering that the deviation of consistency may be caused by random reasons, when testing whether the judgment matrix has satisfactory consistency, it is necessary to compare the CI and the random consistency index *RI* to obtain the test coefficient *CR*, as shown in formula (6):

(6) $$\begin{array}{c} CR=\frac{CI}{RI}. \end{array}$$

Generally, if *CR* < 0.1, it is considered that the judgment matrix passes the consistency test; otherwise, it does not have satisfactory consistency.

In practice, the following method can be used to calculate the approximation of the maximum eigenvalue *λ*max (*A*) of the pairwise comparison matrix 4 = (*aij*) and the corresponding eigenvector. Definition formula (7):

(7) $$\begin{array}{c} U_{k}=\frac{\sum_{j=1}^{n}a_{kj}}{\sum_{i=1}^{n}\sum_{j=1}^{n}a_{kj}}. \end{array}$$

It can be viewed approximated as the eigenvector of *A* corresponding to the maximum eigenvalue. Calculated formula for (8):

(8) $$\begin{array}{c} \lambda =\frac{1}{n}\sum_{u_{i}}^{n}\frac{{\left(AU\right)}_{i}}{u_{i}}. \end{array}$$

It can be approximated as the maximum eigenvalue of *A*. In practice, we can judge the consistency of the matrix *A*.

## 4. Results

### 4.1. Analysis on Boundary Determination Results of the Park

The final analysis result is obtained by making superposition analysis on the influence factors of every index by using the spatial superposition analysis tool of Arc GS10.1 according to the calculation formula of wetland park boundary suitability index above. It can be seen from the figure that there are five levels of areas. The first level represents the area that should be most included in the wetland park boundary and the degree of Level 1–5 decreases in turn. In this study, the areas shown in Level 1–3 are classified into the management and control scope of wetland park. On the basis of the above, the management and control scope of the Park is defined (Figure 5). According to the statistics, the specific management and control area of the Park is 340 sq.km, including the water area of 92 sq.km [22]. It can be found by comparing the previous ecological redline scope of wetland park that the potential tourism resources along the lake, such as Shuicheng, Shuijie, Dafu Mountain, remaining industrial mines and lakeside villa area, are all included in the management and control boundary of wetland park and a certain buffer space is left from the determined management and control boundary so as to give full play to its leisure and recreation functions under the premise of ensuring the ecological environment. In addition to the abundant wetland natural resources, Changdang Lake region also boasts profound wetland cultural resources, such as the local fishing culture, Confucian culture, Zen culture, and characteristic folk culture, all of which constitute the human ecosystem of Changdang Lake Basin. These wetland cultural resources survive mainly relying on the surrounding traditional villages and towns. The wetland park management and control boundary will bring these villages and towns into the scope of management and control, which is conducive to the protection and inheritance of Changdang Lake wetland cultural resources, and promotes the formation of a multicomponent ecological safety pattern of the Park's natural ecology and human ecology; 15% of the water area of Changdang Lake within the jurisdiction of Liyang City is included in the management and control boundary of the Park. So far, the entire water area of Changdang Lake is included within the management and control boundary of the wetland park, which fully guarantees the integrity of the wetland ecosystem of Changdang Lake and facilitates the healthy and sustainable development of the Park's wetland ecosystem.

### 4.2. Boundary Determination and Protection Strategy of the Park

#### 4.2.1. Integrate the Natural and Human Ecological Resources in the Lake Basin

The main purpose of lake-type wetland park construction is to protect lake wetland ecological resources and promote the healthy and sustainable development of lake wetland ecosystem. Wetland ecological resources mainly include natural and human ecological resources. Therefore, it is imperative to integrate the wetland natural and human ecological resources along the lake and its basin scope or within the scope of influence, break the restrictions of administrative divisions, and build the wetland ecological security pattern combining the whole lake basin's natural and human ecology on the basis of the lake when determining the management and control boundary of lake-type wetland park.

#### 4.2.2. Build Two-Layer Wetland Boundary Protection System

The lake ecosystem refers to the wetland ecological environment protection system built through the interaction of wetland park management and control boundary and ecological redline based on the ecological characteristics of the lake-type wetland park ecosystem. The ecological red line of Lake-type wetland park is mainly controlled by rigidity. The ecological redline of lake-type wetland park should be managed mainly by compulsory means and lake wetland ecological conservation activities are forbidden within the management and control scope. It is allowed to build a small number of auxiliary facilities on the basis of not damaging the natural ecological environment of wetland to meet the multi-functional benefits of the wetland park. It is strictly prohibited to carry out activities unrelated to wetland ecological protection, leisure and tourism, science popularization, education, etc [23]. The management and control boundary of Wetland Park is mainly to ensure the dynamic and sustainable integrity of the ecological space in the lake area. The flexible management and control boundary is defined by considering the influencing factors of boundary determination systematically and comprehensively based on the landscape ecology theory.

#### 4.2.3. Build Dynamic Supervision System in Boundary Area

Two different development demands have been proposed in the areas on both sides of the management and control boundary, that is, the internal needs of the wetland park for protecting wetland ecological environment and resources and the area beyond the management and control boundary for meeting the production and service needs of the local residents and tourists [24]. The two kinds of demands interact with each other and show periodic changes with the development of wetland park. Therefore, the management and control boundary line of wetland park always changes. It is necessary to build a dynamic regulatory system for the boundary area of wetland park in order to ensure wetland park's internal ecosystem integrity and reduce the interference of external human factors on wetland park's internal ecological environment. The boundary area of wetland park can be supervised dynamically using geographic information technology and remote sensing technology that have been developed, in order to regulate and control human activities from the very beginning.

## 5. Discussion

Wetland park serves as a key carrier to protect wetland resources. Scientific and reasonable determination of wetland park management and control boundary plays a basic role in ensuring the sustainable development of wetland ecological environment. In this paper, AHP is introduced into the process of multiinfluencing factor analysis of GIS technology so as to fully exert the advantages of GIS technology by combining the strength of both, such as high speed and efficiency, data superposition, and the combination of AHP multi-criteria and quantification, so as to strike a balance between subjectivity and objectivity. The above improves the operability and scientificity of wetland park boundary determination dramatically.

Wetland park should be developed by considering its ecological effect as well as the socioeconomic effect and efforts should be made to give full play to its ecological value, aesthetic value, and socioeconomic value. The study of the previous researches on wetland boundary determination is mostly from the perspective of physical geography and ecology. The determination index and wetland type are single and lack of timeliness, which is difficult to meet the functional requirements of wetland park that integrates ecological protection, ecotourism, science popularity, and education. Wetland resources mean a lot to maintain wetland park's vitality and tourists' most intuitive perception of wetland resources is mainly realized by vision. Dominated by the conventional thinking of “ecological protection,” the traditional boundary determination method ignores the landscape visual value of wetland resources, and splits the regional cultural continuity and socioeconomic relevance between wetland park and surrounding areas. From the perspective of landscape architecture, this study introduces two decisive factors, that is, vision and human geography, from ecological level, and takes into account the comprehensive benefits of wetland park, making wetland park boundary determination more scientific and reasonable.

As a complex and huge ecosystem with high ecological diversity and species diversity, wetland carries out various energy exchanges and material circulations with its surrounding areas, so the influencing factors of wetland park boundary determination are also complex and diverse. Three project layers and 12 index layers are selected in this paper. In the follow-up study, relevant knowledge of various disciplines can be further integrated to enrich the influence index factors of wetland park boundary determination, so as to make boundary determination more accurate and scientific and ensure the sustainable development of wetland biological resources. This study provides a new idea to determine the management and control boundary of wetland park from an interdisciplinary perspective. Taking Changdang Lake National Wetland Park as an example, this paper builds the determination system of management and control boundary of lake-type wetland park preliminarily. This kind of boundary determination system, which combines GIS technology with AHP, is suitable for the determination of not only lake-typed wetland park but also other types of wetland park boundary determinations through adjusting the specific index influence factors as appropriate. It can also provide reference for other nature reserves boundary determination so as to promote the sustainable development of global ecological resources.

## 6. Conclusion

This study combines GIS technology and AHP to remove the errors ascribed to a single method effectively and avoid the dependence on experts' subjective evaluation method and the unavailability of objective data. From the perspective of landscape architecture and landscape ecology, 12 subindicators are selected from three levels including visual control, human geography, and ecological control by combining GIS technology and satellite remote-sensing information with AHP, so as to build the Park's boundary determination system and define the Park's boundary control scope. The newly determined management and control boundary is square kilometers, which effectively solves a series of problems ascribed to the previous boundary determination based on water surface, roads, farmland, and administrative boundaries, such as the lack of dynamic regulation of lake area, the imbalance of the ecosystem protection of lake area, and the disconnection of development for the areas surrounding the lake area. The following requirements for boundary determination and management and control of the Park are proposed as follows according to the determination results: integrate the natural and human ecological resources of the lake basin; build dual-layer boundary management and control system of wetland as well as three strategies for the dynamic regulatory system of boundary area in order to guide the sustainable development of wetland resources.

## Figures and Tables

**Figure 1:** Location of the study area.

**Figure 2:** The images of current boundary of Changdang Lake National Wetland Park.

**Figure 3:** The images of the factor analysis result: (a) road vision; (b) scene source vision; (c) visual sensitivity of relative slope landscape; (d) visual sensitivity of relative distance landscape; (e) elevation; (f) slope; (g) scene source grade; (h) village and town construction; (i) road traffic; (j) water conservation; (k) soil conservation; (l) vegetation.

**Figure 4:** The images of project layer. (a) Visual control, (b) Human geography factor, (c) Ecological control.

**Figure 5:** The image of management and control scope of Changdang Lake National Wetland Park.

**Table 1:** Boundary determination index system.

Target Layer	Project Layer	Index Layer	Indicator Attribute
Boundary determination	Visual control	Road vision	Degree of visible landscape area of road
		Scene source vision	Degree of visible landscape area of scenic spot
		Visual sensitivity of relative slope landscape	Landscape visibility of different slopes
		Visual sensitivity of relative distance landscape	Landscape visibility at different distances
	Human geography factors	Elevation	The relief of the terrain
		Slope	The steepness of the terrain
		Scene source grade	Distance from scene source
		Village and town construction	Buffer distance from town/Village
		Road traffic	Buffer distance from expressway/National and provincial highways
	Ecological control	Water conservation	Distance from water body
		Soil conservation	Land type
		Vegetation	Vegetation coverage

**Table 2:** 9 level Scale.

Scale	Meaning
1	Indicates that the two factors are of the same importance
3	The former is slightly more important than the latter
5	The former is significantly more important than the latter
7	The former is intensely more important than the latter
9	The former is extremely more important than the latter
2, 4, 6, 8	Indicates the median of the above adjacent judgments

**Table 3:** Index weight and classification standard.

Target Layer	Project Layer (Weight)	Index Layer (Weight)	Classification Standard				
			1	2	3	4	5
Boundary determination	Visual control (0.3621)	Road vision (0.0973)	<50 m	50–100 m	100–250 m	250–550 m	>550 m
		Scene source vision (0.0934)	<200 m	—	200–400 m	—	>1000 m
		Visual sensitivity of relative slope landscape (0.0753)	<14.5°	—	14.5–30°	—	>30°
		Visual sensitivity of relative distance landscape (0.0961)	<50 m	50–100 m	100–300 m	300–600 m	>600 m
	Human geography factor (0.3501)	Elevation (0.0426)	＞30 m	10–30 m	5–10 m	−5–5 m	<−5 m
		Slope (0.0534)	<3°	3–8°	8–15°	15–30°	>30°
		Scene source level (0.0963)	<300 m	300–500 m	500–1,000 m	1,000–3,000 m	>3000 m
		Village and town construction (0.0735)	>2,000 m/>500 m	1,500–2,000 m	1,000–1,500 m 250–500 m	500–1,000 m	<500 m/<250 m
		Road traffic (0.0843)	>3,000 m/>2,000 m	2,000–3,000 m/1,500–2,000 m	1,500–2,000 m/1,000–1,500 m	1,000–1,500 m/500–1,000 m	<1,000 m/<500 m
	Ecological control (0.2878)	Water conservation (0.1026)	<30 m/<20 m	30–50 m	50–100 m/20–50 m	100–200 m	>200 m/>50 m
		Soil conservation (0.0875)	Forest land and water area	Cultivated land and garden land	Grassland and unused land	Traffic land	Residential area and industrial and mining land
		Vegetation (0.0977)	>0.4	0.3–0.4	0.2–0.3	0.1–0.2	<0.1

## Data Availability

The data used to support the findings of this study are available from the corresponding author upon request.
